# Clinical sequelae of the novel coronavirus: does COVID-19 infection predispose patients to cancer?

**DOI:** 10.2217/fon-2020-0300

**Published:** 2020-05-27

**Authors:** Priya Hays

**Affiliations:** ^1^Principal, San Mateo, CA 94402, USA

**Keywords:** clinical sequelae, consequences of infection, COVID-19, global pandemic, innate and adaptive immune response, novel coronavirus, oncology, SARS-CoV-2

## Abstract

As cancer patients are clinically known to be predisposed to COVID-19 infection, a corollary question of whether COVID-19 infection predisposes to cancer is explored. This article seeks to establish an association between novel coronavirus sequelae and cancer. A literature review on COVID-19 mechanisms of action, molecular responses it elicits upon infection and tumorigenesis pathways is conducted to establish this association. Major signaling pathways implicated in aberrant cellular growth are activated, the ensuing cytokine storm weakens the immune system response to tumors, and patients may develop cancer as a result of superimposed mutagenic and/or carcinogenic events. Future work needs to be performed to support this hypothesis, both in *in vitro* models and preclinical studies. COVID-19 patients may need to be monitored post-infection for developing cancer.

The novel coronavirus, and the COVID-19 infection it causes, has led to a global pandemic. From its first cases in Wuhan, China in December 2019, it has spread to Italy, Spain and now the USA, among other countries, with devastation. A robust scientific and medical literature emerged to provide information on patients vulnerable to succumbing to the infection. Clinicians warned that cancer patients were particularly susceptible to the novel coronavirus and they, along with their treating oncologists, should remain vigilant [1]. Lung cancer patients are especially forewarned and should be the priority group for COVID-19 prevention. The protection provisions and control measures aiming to protect lung cancer patients from COVID-19 pose increasing concerns [1]. During the COVID-19 outbreak period, differential diagnosis for fever and respiratory symptoms for lung cancer patients receiving antitumor treatment should take place, in order to evaluate the risk of COVID-19 [1]. Moreover, it is necessary to carry out meticulous and individualized clinical management for lung cancer patients to effectively protect the patients from COVID-19 [1]. Additionally, the American Society of Clinical Oncology released a series of statements urging appropriate care for oncology patients at risk for viral infection, and to treat cases with caution (email communication).

This review considers a differently posed question: what are the clinical sequelae of patients who are infected with the novel coronavirus and what medical problems might they face in the future post-infection? These patients are now faced with pneumonia, tissue damage and even multiple organ failure. While these symptoms may lead to morbidity, there is an asymptomatic population who will recover that may possess more health conditions. Even those who have mild-to-moderate clinical presentation may be at risk for other illnesses. The focus in this article is on oncology, and is timely since the virus mediates an immune response, weakens the immune system and causes inflammation, and genetically enters and lyses host cells, and releases its genome into the cytoplasm. According to a recent review, long-term complications among survivors of infection with SARS-CoV-2 having clinically significant COVID-19 disease are not yet available, however, the mortality rates for cases globally remain between 1 and 2% [2]. While this currently remains the case, along with considering some of the future clinical consequences of being infected with SARS-CoV-2, this article calls for subsequent studies into what remains in store for this distinct health population especially with regards to oncology.

## COVID-19 infection: epidemiology & clinical presentation

As of 28 April 2020, worldwide there were more than 2.9 million confirmed cases of COVID-19 with a mortality of about 203,000. In the USA, there were more than 968,000 confirmed cases of COVID-19 and more than 54,000 deaths [3]. The complete clinical manifestation is not clear yet, as the reported symptoms range from mild-to-severe, and may result in the mortality just indicated [4]. Fever, cough, myalgia or fatigue, pneumonia, and complicated dyspnea are the most commonly reported symptoms; headache, diarrhea, hemoptysis, runny nose and phlegm-producing cough are less commonly reported [4]. Patients with mild symptoms were reported to recover after 1 week while severe cases were reported to experience progressive respiratory failure due to alveolar damage from the virus, which may lead to death [4]. Cases resulting in death were primarily middle-aged and elderly patients with pre-existing diseases (chronic respiratory disease, cancer, tumor surgery, cirrhosis, hypertension, coronary heart disease, diabetes and Parkinson’s disease) [4]. Risk factors include being elderly, having poor immune function, having chronic co-morbidities, long-term usage of immunosuppressive agents and having a prior history of surgery before admission [4]. Case definition guidelines mention the following symptoms: fever, decrease in lymphocytes and white blood cells, new pulmonary infiltrates on chest radiography, and no improvement in symptoms after 3 days of antibiotics treatment [4]. Our understanding of co-morbidities and risk factors is evolving as clinical data emerges. A recent study in the *Journal of the American Medical Association* considered the characteristics, clinical presentation and outcomes of patients hospitalized with COVID-19 in the USA and found that of 5700 patients hospitalized with COVID-19 in the New York City area, the most common co-morbidities were hypertension, obesity and diabetes. Among patients who were discharged or died (n = 2634), 14.2% were treated in the intensive care unit, 12.2% received invasive mechanical ventilation, 3.2% were treated with kidney replacement therapy and 21% died [5].

Additionally, heart damage, neurologic symptoms, kidney damage and blood clots have been observed in COVID-19 patients [6]. One review found about 40% of seriously ill COVID-19 patients in China experienced arrhythmias and 20% experienced other cardiac injuries. A separate study of 416 hospitalized COVID-19 patients in China found that 19% showed signs of heart damage, and those patients were more likely to die [7]. According to the study, 51% of patients with heart damage died, compared with 4.5% of patients who showed no signs of cardiac injury [7]. A group of Chinese doctors in another study published found that more than a third of 214 hospitalized COVID-19 patients in Wuhan had neurologic symptoms, the most common of which were dizziness, headaches, impaired consciousness, loss of taste and smell, and skeletal-muscle injuries [8]. More serious but less commonly reported symptoms included seizures and stroke, according to the study [8]. The findings have prompted doctors to begin performing simple neurological exams on COVID-19 patients [6]. Also, early data showed 14–30% of ICU COVID-19 patients in New York and Wuhan, lost kidney function and later required dialysis [6]. Similarly, a study found that nine of 26 people who died of COVID-19 in Wuhan had acute kidney injuries, and seven had units of the new coronavirus in their kidneys [9]. The new coronavirus also appears to produce blood clots that can travel from patients’ veins to their lungs, causing a pulmonary embolism, and other organs [6]. Chinese researchers in one report said they found small blood clots in about 70% of the patients who died of COVID-19 and were included in the study. In comparison, the researchers found similar blood clots in fewer than one in 100 patients who survived the disease [6]. In a separate peer-reviewed study of 81 patients in Wuhan, researchers wrote that 20 patients experienced pulmonary embolism and eight died from the condition [10]. Clinicians and researchers have yet to determine whether the new coronavirus is directly attacking those organs, or whether the injuries are caused by the patients’ immune responses to infection [6]. Additionally, there is variation in recovery in patients and evidence of long-term persistence of the virus that may be etiology of lung inflammation and pneumonitis, and instances of hypoxia. Patients may be predisposed to cancer as a result of the organ damage the virus is associated with.

## Structure & pathophysiology of SARS-CoV-2

As shown in Figure 1, SARS-CoV-2 (CoV)s are enveloped, positive-stranded RNA viruses with a nucleocapsid. For addressing pathogenetic mechanisms of SARS-CoV-2, its viral structure and genome must be considered [2]. In CoVs, the genomic structure is organized in a +ssRNA of approximately 30 kb in length – the largest known RNA viruses – and with a 5′-cap structure and 3′-poly-A tail (Figure 2) [2]. The virus goes from producing its RNA, to the creation of the of polyprotein 1a/1ab (pp1a/pp1ab) in the host [2]. Figure 3 shows how the viral replication-transcription complex is the product of the transcription apparatus which is housed in double-membrane vesicles formed from subgenomic RNAs [2]. Open reading frames serve as templates for the production of the subgenomic mRNAs. In between these open reading frames, transcription termination occurs at transcription regulatory sequences [2]. At least six open reading frames are present, including a frameshift able to block host innate immune response. The viral envelope, a structural protein, confers viral pathogenicity since it promotes viral assembly and release. However, many of these features (e.g., those of nonstructural protein 2, and 11) have not yet been described [2].

**Figure 1.** Structure of SARS-CoV2. A positive single-stranded RNA genome with a nucleocapsid is surrounded by a membrane with spike proteins. Reproduced with permission from [2] © StatPearls (2020).

**Figure 2.** The SARS CoV-2 genomic structure. A papain-like protease, 3CL-protese and endoribonuclease are produced to lyse host cells. The replicase gene codes for replicative apparatus to create more virus to infect host cells. Reproduced with permission from [2], © StatPearls (2020).

**Figure 3.** Coronavirus Infection Course. How the novel coronavirus infects host cells. E: Envelope; ER: Endoplasmic reticulum; M: Membrane; S: Spike. Reproduced with permission from [3].

The spike glycoproteins of CoV are composed of two subunits S1 and S2. The S2 protein is highly conserved and contains a fusion peptide, a transmembrane domain and a cytoplasmic domain [2]. The S subunits consists of homotrimers that compose the spikes on the viral surface which can transduce through host receptors. Thus, it could be a target for antiviral (anti-S2) compounds. On the contrary, the spike receptor-binding domain presents only a 40% amino acid identity with other SARS-CoVs [2]. Other structural elements on which research must necessarily focus are the ORF3b that has no homology with that of SARS-CoVs and a secreted protein (encoded by *ORF8*), which is structurally different from those of SARS-CoV.

Mutations and strain recognitions can be determined from the SARS-CoV-2 gene sequences that were recently published. A spike mutation which may have occurred in late 2019 triggered jumping to humans. In particular, SARS-CoV-2 gene sequence was compared with that of SARS-CoV. They analyzed the transmembrane helical segments in the ORF1ab encoded 2 (nsp2) and nsp3 and found that position 723 presents a serine instead of a glycine residue, while the position 1010 is occupied by proline instead of isoleucine [2]. The matter of viral mutations is key for explaining potential disease relapses.

## COVID-19 infection & the immune response it elicits

### Immune response against the novel coronavirus

The current understanding of how a dysregulated immune response that causes lung immunopathology would lead to deleterious clinical manifestations after pathogenic hCoV infections was reported in prior studies. As early as 2017, Channappanavar and Perlman declared that recent identification of SARS-like coronaviruses in bats and MERS-CoV in domesticated camels makes it likely that these viruses will continue to cross species barriers and cause additional outbreaks in human populations [11]. These highly pathogenic hCoVs cause a wide spectrum of clinical manifestations in humans, with a large fraction of patients developing short period of moderate clinical illness and a small but a substantial number of patients experiencing severe disease characterized by acute lung inflammation and acute respiratory disease [11].

There are certain inflammatory responses that may be conducive to cancer. IFN-α/β or inflammatory monocyte-macrophage-derived pro-inflammatory cytokines sensitized T cells to undergo apoptosis, further impeding virus clearance [11]. The loss of TIR-domain-containing adapter-inducing IFN-β (TRIF), an adapter molecule for TLR-3 and TLR-4 signaling, resulted in a distinct inflammatory signature characterized by neutrophil and other inflammatory cell infiltration [11]. A dysregulated immune response to SARS-CoV in TRIF-deficient mice was associated with aberrant antiviral IFN (IFN-α and IFN-β), pro-inflammatory cytokine and chemokine (IL-6, TNF, IFN-γ and monocyte chemoattractant CCL5), and interferon-stimulated gene (*RSAD2*, *IFIT1* and *CXCL10*) responses, another possible indicator of cancer risk [11].

Multiple structural and nonstructural proteins of SARS-CoV antagonize interferon responses [5]. Very early after infection, hCoV reach high titers and sequester multiple proteins that inhibit the interferon response, suggesting that immune response delay or evasion may be the result of early antagonism of the interferon [11]. A dysfunctionally regulated inflammatory response and T-cell apoptotic sensitization is also further orchestrated by the delayed interferon signaling [11].

Some consequences of cytokine storm and immunopathology are epithelial and endothelial cell apoptosis and vascular leakage, suboptimal T-cell response, in other words. CoV-specific T cells are crucial for virus clearance and limit further damage to the host. Additionally, T-cell responses also dampen overactive innate immune responses [11]. Exuberant inflammatory responses caused by pathogenic hCoV diminish the T-cell response, in the case of SARS CoV infection via TNF-mediated T-cell apoptosis, thus resulting in uncontrolled inflammatory response; accumulation of alternatively activated macrophages and altered tissue homeostasis; and acute respiratory distress syndrome [11].

Figure 4 demonstrates the enormous immune response against the novel coronavirus [12]. The innate immune response and adaptive immunity have distinct responses to coronaviruses infection [12]. The SARS-Cov-2 (CoV) infects macrophages, and then macrophages present CoV antigens to T cells and this process leads to T-cell activation and differentiation, including the production of cytokines associated with the different T-cell subsets (i.e., T helper cells), followed by a massive release of cytokines for immune response amplification [12]. The continued production of these mediators due to viral persistence has a negative effect on natural killer cells and CD8^+^ T-cell activation, and CD8^+^ T cells produce very effective mediators to clear CoV [6].

**Figure 4.** COVID-19 infection and the immune response. Activated signaling pathways such as JAK–STAT and MAPK, cytokine storm, T-cell depletion, humoral responses and high levels of inflammation may predispose patients infected with novel coronavirus to cancer. Reproduced with permission from [12].

The attachment of CoV to DPP4R on the host cell through S protein leads to the appearance of genomic RNA in the cytoplasm. An immune response to dsRNA that results can be partially generated during CoV replication. TLR-3 sensitized by dsRNA leads to cascades of signaling pathways (IRFs and NF-κB activation, respectively) which are activated to produce type I interferons and pro-inflammatory cytokines [12]. The production of type I interferons is important to enhance the release of antiviral proteins for the protection of uninfected cells. Sometimes, accessory proteins of CoV can interfere with TLR-3 signaling and bind the dsRNA of CoV during replication to prevent TLR-3 activation and evade the immune response [12].

TLR-4 might recognize S protein and lead to the activation of pro-inflammatory cytokines through the MyD88-dependent signaling pathway. Virus–cell interactions lead to the strong production of immune mediators [6]. The secretion of large quantities of chemokines and cytokines (IL-1, IL-6, IL-8, IL-21, TNF-β and MCP-1) is promoted in infected cells in response to CoV infection. These chemokines and cytokines, in turn, recruit lymphocytes and leukocytes to the site of infection [12].

## Novel coronavirus & oncologic sequelae: how cancer may be implicated

The host innate immune system detects viral infections by using PRRs to recognize pathogen-associated molecular patterns (PAMPs). At present, the known PRRs mainly include TLR, RIG-I-like receptor, NOD-like receptor, C-type lectin-like receptors and free-molecule receptors in the cytoplasm, such as cGAS, IFI16, STING and DAI [12].

PAMPs recognized by TLRs include lipids, lipoproteins, proteins and nucleic acids of the bacterial, viral, parasite and fungal origins [12]. The recognition of PAMPs by TLRs also occurs in cell membranes, endosomes, lysosomes and endocyte-lysosomes and other locations in cells [12]. Different TLRs can induce different biological responses via subsequent activation of varied adapter proteins, such as MyD88, TIRAP, TRIP and TRAM, but these adapter proteins all share the TIR structure [12].

Viral infection plays a key role in signaling factor activation, that may have relevance for the initiation of cancer. MyD88 is the first identified TIR family member, which acts as an adapter protein; it mainly activates the transcription factors NF-κB and MAPKs pathways to induce inflammatory factors expression [12]. Additionally, after a TLR is activated by the corresponding PAMP, MyD88 recruits the receptor-related kinases IRAK4, IRAKI, IRAK2 and IRAK-M. IRAK4 plays an important role in activating NF-κB and MAPKs downstream of MyD88. IRAK interacts with TRAF6, which causes its K-63 ubiquitination, and facilitates NEMO ubiquitination to activate NF-κB, which may have implications for aberrant cell growth. TRIF-dependent pathways activate IRF3 and NF-κB. The function of TRAM and TIRAP is to recruit TRIF molecules to the TLR4 receptor and MyD88 to the TLR2 and TLR4 receptors, promoting cellular growth [12].

Other signaling pathways are activated. Depletion of CD4^+^ T cells is associated with reduced pulmonary recruitment of lymphocytes and neutralizing antibody and cytokine production, resulting in a strong immune-mediated interstitial pneumonitis and delayed clearance of SARS-CoV from lungs [12]. Additionally, T helper cells produce pro-inflammatory cytokines via the NF-κB signaling pathway. IL-17 cytokines recruit monocytes and neutrophils to the site of infection with inflammation and activate other downstream cytokine and chemokine cascades, such as IL-1, IL-6, IL-8, IL-21, TNF-β and MCP-1 [12].

There may be a distinct association between novel coronavirus infection and the onset of cancer through the activation of the MAPK and JAK–STAT signaling pathways and the NF-κB transcription factor. The MAPK signaling pathway, activated upon COVID-19 infection, is involved in the tumorigenesis of a number of cancers, including hepatocellular carcinoma, adrenocortical cancer, endometrial cancer, colorectal cancer and pituitary adenomas. The Ras/MAPK pathway is activated in 50–100% of human hepatocellular carcinomas and is correlated with a poor prognosis [13]. The MAPK signaling pathway is also implicated in pituitary adenomas and because of the important roles of MAPK signaling pathways in tumorigenesis, the use of the MAPK signaling pathways as therapeutic targets has continuously been considered as a promising strategy for pituitary adenoma therapy [14]. In the context of the role of two of the MAPK signaling pathways (ERKs 1/2 and p38), data suggest that MEK-MAPK-ERK signaling has a role in adrenocortical tumorigenesis that could be potentially used as a diagnostic marker for malignancy and targeted treatment in adrenocortical carcinoma [15]. Cholesterol in the form of LDL enhances intestinal inflammation and colorectal cancer progression via activation of reactive oxygen species (ROS) and signaling pathways including the MAPK pathway; [16] and, the estrogen receptor-α activates MAPK signaling pathway to promote the development of endometrial cancer [17]. The oncologic sequelae of COVID-19 may include these cancers upon viral activation of the MAPK signaling pathway. These tumorigenic pathways may play a role in cancer initiation and progression in COVID-19 infection.

The JAK–STAT signaling pathway is also activated by type I interferon synthesis promoted by IRF3 and IRF7 activation. This has been through PRRs that recognize viral RNA. The activation JAK–STAT signaling pathway has shown to be involved in tumorigenesis, including T-cell lymphoma, lung cancer and breast cancer. Gene expression profiling has implicated several intracellular signaling cascades, including the JAK/STAT pathway, in the pathogenesis of particular subtypes of lymphoma [18]. JAK–STAT signaling pathways are mutationally activated in many extranodal T-cell lymphomas, such as natural killer/T-cell and hepatosplenic T-cell lymphomas [19]. Since the JAK–STAT pathway is considered to be a central player in inflammation-mediated tumorigenesis, the implication of JAK–STAT signaling and the therapeutic potential of JAK1/2 inhibition was investigated in K-RAS-driven lung adenocarcinoma, and data showed that JAK1 and JAK2 are activated in human lung adenocarcinoma and that increased activation of JAK–STAT signaling correlated with disease progression and K-RAS activity in human lung adenocarcinoma [20]. Dysregulated JAK/STAT signaling has been implicated in breast cancer metastasis, which is associated with high relapse risks, which may be mediated through *GRAM1b* [21].

NF-κB, and TRIF-dependent pathways are also activated; and, IRF3 and IFN-β are activated in turn [12]. Transcription factors IRF3 and NF-κB induce the gene expression of type I interferon through their activation by adaptor protein TRIF of TLRs. TLRs classify these types of signaling pathways induced by viral infection: The TLR signaling pathways are classified as the MyD88-dependent pathway, which functions to activate immune inflammatory factors and the TRIF-dependent pathway, which then in turn functions to activate the type I interferons and inflammatory factors [12]. NF-κB-driven gene products include cytokines/chemokines, growth factors, anti-apoptotic factors, angiogenesis regulators and metalloproteinases, and drive oncogenesis. For instance, many of the genes transcribed by NF-κB promote gastric carcinogenesis. Since it has been shown that chemotherapy-caused cellular stress could elicit activation of the survival factor NF-κB, which leads to acquisition of chemoresistance, the NF-κB system is recommended for therapeutic targeting [22]. Prosaposin, a neurotrophic factor, promotes the proliferation and tumorigenesis of glioma through TLR4-mediated NF-κB signaling pathways [23].

Dendritic cells (DCs) also respond to the virus, and their differentiation from precursor cells to mature cells may be inhibited as is the case with HIV-1. If their maturation is blocked, by perhaps the lack of GM-CSF, IL-4 and TNF-α, the adaptive immune response, which plays a key role in the cancer-immunity cycle may be inhibited (Figure 5). DC’s are the major antigen-presenting cells in the organism, and contribute both types of immunity by activating T cells and B cells. Immature DCs have strong migration ability, and mature DCs can effectively activate T cells in the central link of start-up, regulation and maintenance of immune responses [6]. Thus, if the maturation process of DCs is blocked, it directly affects the initiation of subsequent adaptive immune responses that may need to be mobilized in attacking cancer.

Other types of viruses have ostensible effects on adaptive immunity. In the case of HIV-1, DC precursor cells cannot differentiate into DCs if transfected with HIV-1 Nef protein in the presence of the inducers, indicating that Nef blocks the differentiation of DC precursor cells into mature DCs [12]. Additionally, both the core protein and NS3 protein of HCV inhibits the expression of CD1a, CD1b and DC-SIGN molecules on human peripheral blood mononuclear precursor cells, which play an important role in the development of peripheral blood mononuclear precursor cells to DCs [12]. In addition, HIV-1 attenuates the MHC I on the surface of DCs, thereby reducing the ability of DCs to present the viral antigens. HIV-1 infection enhances the expression of DC-specific intercellular adhesion molecule-3-grabbing nonintegrity (DC-SIGN), thus inhibiting CC chemokine receptor 7 and MHC-II, which are important receptors of DC homing [12]. These results indicate that virus infection interferes with the differentiation and function of DCs, hinders the subsequent adaptive immune response mediated by DCs and makes the virus evade the adaptive immune response of the host successfully [6]. If these DC events are occurring, cancer may co-opt normal cellular function and evade immune responses in a viral infection such as COVID-19.

A ‘cytokine storm’, an excessive immune reaction in the host, also results from viral mechanisms that results in extensive tissue damage, mediated by IL-produced by activated leukocytes. B lymphocyte differentiation, cell growth stimulation and pathogenesis of some types for cancer may result. These effects are linked to the function of structural and nonstructural proteins of the virus [2]. Cytokine release syndrome, an immune-related adverse effect of chimeric antigen receptor T-cell therapies, is also implicated in the potential emergence of cancer. Additionally, as tissue damage envelopes the body’s physiological functioning, and cellular resources are increasingly devoted to compensating for it, cancer may emerge as a risk factor. Lung tissue damage, a prevalent and major consequence of infection, may be particularly at risk for developing into lung cancer, and patients who experience these symptoms, may need to be monitored for these sequelae.

## Relevance of the cancer-immunity cycle & tumor microenvironment

In the cancer-immunity cycle (Figure 5), the cancer presents antigens which antigen-presenting cells present to MHC to activate cytotoxic CD8^+^ T cells, to ultimately destroy cancer cells in a cyclic process [24]. In cancer, the cancer-immunity cycle is dysfunctional with the accumulation of inhibitors of T-cell response and promoters of cancer cell growth. In SARS-CoV infection, cytotoxic T cells play a significant role and combat the pathogen by killing viral-infected cells and promoting the production of virus-specific antibodies by activating T-dependent B cells. The inflammation observed in the pulmonary environment upon viral infection is due to this large role played by CD8^+^ T cells which lead to immune injury. Immunosuppression, a risk factor for novel coronavirus, may emerge, conversely, as a risk for cancer in the context of viral infection.

**Figure 5.** The cancer-immunity cycle. Dendritic cells present cancer antigens to T cell, which are honed to the cancer site. T cells infiltrate tumors and recognize cancer cells upon their destruction. Each point in this cycle may be points of vulnerability upon novel coronavirus infection. APC: Antigen-presenting cell. Reproduced with permission from [24].

From an understanding of the cancer-immunity cycle, are there are any elements of novel coronavirus infection that would make the cycle vulnerable to cancer at any point and prevent the generation of immunity to cancer? The presence of checkpoint inhibitors to immune responses, such as cytotoxic T-lymphocyte associated protein-4, programmed death-1 and programmed death-ligand-1, may inure the development of cancer with viral infection. In a depleted T-cell environment postinfection, the broad T-cell response to cancer may be undermined. This inflammatory response concomitant with immune cell depletion, whether temporary or not, may lead to oncologic sequelae if accompanied by a superimposed mutagenic and/or carcinogenic event potentially occurring in a time-adjacent manner. Figure 6 displays the tumor microenvironment in the context of breast cancer and illustrates major inflammation and cytokine release, marks of viral infection which may predispose to cancer.

**Figure 6.** Tumor microenvironment of breast cancer. The tumor microenvironment progresses through cytokine release. Reproduced with permission from [25].

## Somatic mutations, drug resistance & COVID-19

The implications for novel coronavirus infection on genomic variability are unknown at this point. If the virus through its replicative [26] and recombination capabilities [27] leads to genetic alterations that may predispose to cancer, another risk factor may be revealed.

The administration of antiviral agents and other proposed treatments such as the antimalarial drug hydroxychloroquine may induce drug resistance to cancer therapies, such as targeted agents and immunotherapies. Even further, the status of targeted therapies may be jeopardized by the infection of the virus, since many personalized agents target growth factors that are possibly affected by viral transduction; however, this remains to be investigated.

## Countervailing viewpoints

It is generally known that viruses can cause cancer by integration of the genomes into host cell chromosomes and the expression of oncoproteins. While both of these mechanisms are not implicated in SARS-CoV-2, these are not exclusive mechanisms. The turning on of oncogenic signaling pathways and the acute inflammatory response that results upon coronavirus infection can be hypothesized as being cancer inducing, or leading to the risk of developing cancer, especially if the patient has a superimposed mutagenic or carcinogenic event occurring concomitantly, even if the virus does not cause a chronic infection like viruses such as HCV, HCV and EBV. Additionally, there exist limited resources and research as a result of the pandemic that may damage the prognosis of cancer patients. Novel coronavirus can destroy T cells, but unlike HIV, does not lead to persistent infection of T cells. Data suggest however that there is a general depletion of T cells in the COVID-19 infection environment, and this may affect the healthy progression of the cancer-immunity cycle. Also, there exist gaps in current knowledge on the novel coronavirus’ impact on the immune system during co-infection by other viruses, such as HCV, HIV and EBV. Finally, the overwhelming organ dysfunction that novel coronaviruses results in some cases should be further investigated, and as possibly having an association with cancer. These should remain areas of research for future study.

## Future perspective

As the population infected with the novel coronavirus grows, and the infection spreads, its clinical sequelae may pose an issue of concern for physicians, and oncologists in particular. Future studies should focus on the predisposition of these recovering patients for cancer, and if these patients need to be monitored for the disease. It is the cumulative effect of many distinguishable aspects of coronavirus infection that leads to the increased predisposition to cancer, which then warrants closer follow-up in the future. The organ damage, inflammatory response and signaling pathways activation that occur upon viral infection may sum to significantly increase patients’ predisposition to cancer, and this may be compounded by a superimposed mutagenic or carcinogenic event. The oncology field may evolve by investigating the potential tumor microenvironment in the context of SARS-CoV-2 infection, and if the virus can be considered an etiological agent in the development of cancer. Clinical sequelae may involve physicians needing to refer COVID-19 cases to oncologists for the confirmation of cancer, either benign and malignant cases. The caveat must be mentioned however that knowledge surrounding coronavirus is constantly being updated and this review must be interpreted in light of any recently updated knowledge.

**Executive summary**

- The novel coronavirus is leading to a global pandemic and is causing worldwide clinical and economic devastation. The infection may pose medical risk factors for patients, both symptomatic and asymptomatic, who recover. There will be a distinct health population in the future that will need to deal with clinical sequelae, and cancer may be one of them.

**Oncologic sequelae of the novel coronavirus**

- Viral infection induces a robust immune response, a ‘cytokine storm’ leading to tissue damage and inflammation, which may predispose to cancer. Signaling factors, such as MAPK and JAK–STAT, promoted by viral infection may lead to aberrant cellular growth that marks cancer. The maturation of dendritic cells may be inhibited, as shown in patients infected with HIV-1.

**The cancer-immunity cycle & tumorigenesis**

- The cancer-immunity cycle may be impaired upon viral infection, since T-cell apoptosis also occurs as a result of viral infection, leading to a state of immunosuppression. If concomitant with a mutagenic or carcinogenic event, a cancerous state may result. The ‘cytokine storm’ poses a risk factor for cancer in the tumor microenvironment.

**Summary**

- In conclusion, patients infected and recovered from novel coronavirus, particularly those with lung tissue damage, may need to be monitored for cancer, among other diseases.
